The article "Anti-inflammatory adipokines: chemerin, vaspin, omentin concentrations and SARS-CoV-2 outcomes" was published in 2021. Journal: Sci Rep.

# Anti-inflammatory adipokines: chemerin, vaspin, omentin concentrations and SARS-CoV-2 outcomes

**DOI:** 10.1038/s41598-021-00928-w

**Published:** 2021-11-02

**Authors:** Michał Kukla, Tomasz Menżyk, Marcin Dembiński, Marek Winiarski, Aleksander Garlicki, Monika Bociąga-Jasik, Magdalena Skonieczna, Dorota Hudy, Barbara Maziarz, Beata Kusnierz-Cabala, Lubomir Skladany, Ivica Grgurevic, Małgorzata Wójcik-Bugajska, Tomasz Grodzicki, Dominika Stygar, Tomasz Rogula

**Affiliations:** 1 Department of Internal Medicine and Geriatrics, Faculty of Medicine, Jagiellonian University Medical College, Cracow, Poland; 2 Department of Endoscopy, University Hospital in Kraków, Cracow, Poland; 3 Department of Internal Medicine, Gastroenterology and Acute Intoxication, Regional Hospital, Tarnów, Poland; 4 2nd Department of General Surgery, Faculty of Medicine, Jagiellonian University Medical College, Cracow, Poland; 5 Chair of Gastroenterology, Hepatology and Infectious Diseases, Faculty of Medicine, Jagiellonian University Medical College, Cracow, Poland; 6 Department of Systems Biology and Engineering, Silesian University of Technology, 44-100 Gliwice, Poland; 7 Biotechnology Centre, Silesian University of Technology, 44-100 Gliwice, Poland; 8 Chair of Clinical BioChemistry, Department of Diagnostics, Faculty of Medicine, Jagiellonian University Medical College, 31-501 Cracow, Poland; 9 Department of Internal Medicine and HEGITO (Hepatology, Gastroenterology and Liver Transplantation), F.D. Roosevelt University Hospital, Banska Bystrica, Slovakia; 10 Zagreb University School of Medicine, Šalata ul. 2, 10000 Zagreb, Croatia; 11 Division for Liver Diseases, Department of Gastroenterology, Dubrava University Hospital, Zagreb, Croatia; 12 Department of Physiology, School of Medicine with the Division of Dentistry in Zabrze, Medical University of Silesia, 40-055 Katowice, Poland; 13 Case Western Reserve University School of Medicine, Cleveland, OH USA; 14 1st Department of General Surgery, Faculty of Medicine, Jagiellonian University Medical College, Cracow, Poland

**Keywords:** Prognostic markers, Infection, SARS-CoV-2

## Abstract

Coronavirus disease 2019 (COVID-19) is associated with systemic inflammation. A wide range of adipokines activities suggests they influence pathogenesis and infection course. The aim was to assess concentrations of chemerin, omentin, and vaspin among COVID-19 patients with an emphasis on adipokines relationship with COVID-19 severity, concomitant metabolic abnormalities and liver dysfunction. Serum chemerin, omentin and vaspin concentrations were measured in serum collected from 70 COVID-19 patients at the moment of admission to hospital, before any treatment was applied and 20 healthy controls. Serum chemerin and omentin concentrations were significantly decreased in COVID-19 patients compared to healthy volunteers (271.0 vs. 373.0 ng/ml; *p* < 0.001 and 482.1 vs. 814.3 ng/ml; *p* = 0.01, respectively). There were no correlations of analyzed adipokines with COVID-19 severity based on the presence of pneumonia, dyspnea, or necessity of Intensive Care Unit hospitalization (ICU). Liver test abnormalities did not influence adipokines levels. Elevated GGT activity was associated with ICU admission, presence of pneumonia and elevated concentrations of CRP, ferritin and interleukin 6. Chemerin and omentin depletion in COVID-19 patients suggests that this adipokines deficiency play influential role in disease pathogenesis. However, there was no relationship between lower adipokines level and frequency of COVID-19 symptoms as well as disease severity. The only predictive factor which could predispose to a more severe COVID-19 course, including the presence of pneumonia and ICU hospitalization, was GGT activity.

## Introduction

The pathogen causing the coronavirus disease 2019 (COVID-19) is severe acute respiratory syndrome coronavirus 2 (SARS-CoV-2), an enveloped RNA virus. Human SARS-CoV-2 infection leads to a variety of manifestations that include the asymptomatic carrier status, acute respiratory disease (ARD), and pneumonia^1^. On March 11, 2020, the WHO declared this outbreak a Pandemic, since it affected more countries and threatened the lives of patients worldwide^2^. Since the outbreak of COVID-19 different digestive symptoms have also been frequently reported in infected patients^3,4^.

Several studies have documented metabolic disorders to be associated with not only increased risk of SARS-CoV2 infection but primarily with worse prognosis and as a consequence higher mortality rates. Obesity, defined as body mass index (BMI) ≥ 30 kg/m^2^, is a risk factor for mortality in COVID-19. Patients with concomitant obesity are more likely to develop a critical illness^5,6^. Furthermore, it has been shown that most of the SARS-CoV-2 infected patients that are admitted to the intensive care unit with respiratory failure who need advanced respiratory support are overweight^7^. A recent study proved that high visceral fat (VF) content is a stronger predictor of severe forms of COVID-19 in non-obese Caucasian patients than BMI or subcutaneous fat, which could be directly associated with pro-inflammatory adipokines secretion by VF^8^. Since diabetes is one of the most common diseases, it is unsurprising that various studies have been investigating the influence of type 2 diabetes mellitus (T2DM) on the COVID-19 course. Accordingly, patients with diabetes are more likely than healthy people to develop COVID-19 disease and complications such as acute respiratory distress syndrome (ARDS) and even death^9^. Several studies have reported SARS-CoV-2 infection associated with liver injury, which usually presented as a mild or moderate elevation of alanine aminotransferase (ALT)/aspartate aminotransferase (AST)^10^. Pre-existing nonalcoholic fatty liver disease (NAFLD), which represents the hepatic manifestation of metabolic syndrome, may clearly have an impact on COVID-19 severity and outcome. According to recent publications, NAFLD is a significant risk factor for hospitalization for COVID-19^11^. Moreover, NAFLD represents a high risk for severe COVID-19 irrespective of gender, and independent of metabolic syndrome specifically in the male gender^12^.

Adipokines are biologically active molecules causing pleiotropic effects. Numerous studies have demonstrated that they are involved in the pathogenesis of metabolic disorders which were mentioned above^13,14^. It is now well established that adipokines have both pro-inflammatory and anti-inflammatory activities. Consequently, dysregulation of adipokine production can have local or systemic effects on inflammatory responses^15^.

Pointing to the essential role of adipokines in metabolic regulation and the immune response we hypothesize that these molecules play an important role in the development and progression of COVID-19. In light of the aforementioned studies, we decided to investigate serum concentrations of three novel adipokines, chemerin, omentin, and vaspin, among patients with SARS-CoV-2 infection. These analyses were performed to assess modifications of adipokine levels among COVID-19 patients in comparison to patients without SARS-CoV-2 infection. We also elucidated the relationship between chemerin, omentin, and vaspin serum levels and COVID-19 severity and concomitant metabolic abnormalities, with emphasis on its correlation with intercurrent liver injury.

## Results

### Baseline characteristics and laboratory data of COVID-19 patients and control group

A total of 70 patients (43 women and 27 men, median age 58.5 [49.0–67.0] years) with COVID-19 proven by RT-PCR were included in the study. Median BMI was 27.8 [25.6–31.4] kg/m^2^.

Serum chemerin and omentin concentrations were significantly decreased in COVID-19 patients compared to healthy volunteers (271.0 [236.4–309.2] vs. 373.0 [363.1–392.3] ng/ml; *p* < 0.001 and 482.1 [327.4–665.2] vs. 814.3 [435.3–1148.5] ng/ml; *p* = 0.01, respectively). There was no significant difference in serum vaspin level between COVID-19 patients and control group (0.16 [0.09–0.28] vs 0.12 [0.09–0.28] ng/ml; *p* = 0.50). Comparing inflammation markers there was no significant difference in white blood cells (WBC) count between these two groups (*p* = 0.06), however considering acute-phase proteins (APPs) there was a significant increase of C-reactive protein (CRP) and especially ferritin among patients with confirmed infection (*p* < 0.001 and *p* < 0.001, respectively). We observed that the ALT and gamma-glutamyl transferase (GGT) activities were significantly higher in COVID-19 patients than in the control group (*p* = 0.02 and *p* = 0.003, respectively), while there were no significant differences in AST activity or bilirubin level (*p* = 0.38 and *p* = 0.25, respectively). Moreover, albumin levels were significantly decreased in infected patients (*p* = 0.02). A detailed comparison of analyzed groups is shown in Table 1.

**Table 1:** The baseline characteristics and laboratory data of patients and healthy volunteers.

Parameters	COVID-19 patients (n = 70)	Healthy volunteers (n = 20)	*p*
Age [years]	58.5 (49.0–67.0)	50.0 (43.0–58.5)	0.02
BMI [kg/m^2^]	27.8 (25.6–31.4)	29.7 (25.3–32.4)	0.67
Chemerin [ng/ml]	271.0 (236.4–309.2)	373.0 (363.1–392.3)	< 0.001
Omentin-1 [ng/ml]	482.1 (327.4–665.2)	814.3 (435.3–1148.5)	0.01
Vaspin [ng/ml]	0.16 (0.09–0.28)	0.12 (0.09–0.28)	0.50
WBC [10^3^/µl]	5.88 (4.51–6.43)	6.78 (5.14–7.49)	0.05
RBC [10^6^/µl]	4.30 (4.07–4.51)	4.66 (4.51–4.99)	0.001
HCT [%]	38.2 (36.4–40.5)	41.5 (39.6–43.4)	0.002
HGB [mg/dl]	12.7 (12.3–13.3)	14.5 (13.2–14.6)	0.001
PLT [10^3^/µl]	246.5 (202.0–333.0)	223.5 (197.0–259.0)	0.17
CRP [mg/l]	5.53 (2.08–18.2)	0.80 (0.50–1.58)	< 0.001
Ferritin [µg/l]	210.0 (114.7–487.0)	16.5 (13.0–19.6)	< 0.001
ALT [IU/l]	34.0 (20.0–52.5)	21.0 (16.0–25.7)	0.02
AST [IU/l]	25.0 (17.5–43.0)	24.0 (20.0–26.5)	0.38
GGT [IU/l]	33.5 (20.0–62.5)	14.0 (10.7–24.2)	0.003
Bilirubin [µmol/l]	6.16 (4.57–8.17)	7.35 (5.40–9.70)	0.25
Fasting glucose [mmol/l]	5.27 (4.70–6.01)	5.50 (4.05–5.73)	0.59
Urea [mmol/l]	5.39 (4.20–6.21)	5.67 (5.45–6.94)	0.16
Creatinine [µmol/l]	66.3 (58.9–87.2)	85.2 (73.3–95.4)	0.01
Cholesterol [mmol/l]	4.80 (3.70–5.57)	5.26 (3.54–6.54)	0.49
Triglycerides [mmol/l]	1.53 (1.26–1.86)	1.83 (1.04–2.03)	0.97
HDL [mmol/l]	1.01 (0.84–1.15)	1.12 (1.06–1.32)	0.12
LDL [mmol/l]	2.48 (1.68–3.32)	2.65 (1.48–4.37)	0.76
INR	0.96 (0.92–1.00)	1.06 (1.00–1.12)	0.009
Total protein [g/l]	65.0 (62.0–71.0)	65.5 (63.0–71.0)	0.75
Albumin [g/l]	40.0 (34.2–43.0)	43.0 (40.0–45.0)	0.02

ALT—alanine transaminase, AST—aspartate transaminase, BMI—body mass index, CRP—C-reactive protein, GGT—gamma-glutamyl-transferase, HCT—hematocrit, HDL—*high-density* lipoprotein, HGB—hemoglobin, INR—international normalized ratio, LDL—low-density lipoprotein, WBC—white blood cells, PLT—platelet count, RBC—white blood cells.

### Comparison between males and females with COVID-19

Serum chemerin, omentin, and vaspin concentrations did not differ significantly between females and males (266.0 [237.9–313.8] vs. 267.4 [234.7–284.0] ng/ml, *p* = 0.47; 435.3 [355.0–681.2] vs. 526.4 [225.4–630.1] ng/ml, *p* = 0.99; 0.17 [0.12–0.29] vs. 0.15 [0.08–0.28] ng/ml, *p* = 0.45, respectively). We also did not observe any significant differences with respect to such inflammation markers as WBC, CRP, procalcitonin (PCT), or interleukin 6 (IL-6). On the other hand, ferritin was significantly lower in men with COVID-19 [176.0 [109.5–351.0] vs. 307.0 [179.0–665.5] µg/l, *p* = 0.04]. Surprisingly, females presented higher ALT levels in comparison to males (42.5 [26.0–61.5] vs. 25.0 [12.5–41.5] IU/l, *p* = 0.01). No significant differences were found in terms of AST, GGT, alkaline phosphatase (ALP), INR, albumin, or iron.

### Comparison of COVID-19 patients with respect to BMI and presence of a metabolic syndrome

The patients were divided into two subgroups based on BMI (BMI < 30 kg/m^2^ and ≥ 30 kg/m^2^). There were no significant differences concerning chemerin, omentin, and vaspin levels in the groups of patients with different BMI (*p* = 0.16, *p* = 0.73, and *p* = 0.30, respectively). There was a significantly higher level of IL-6 among patients with obesity (5.32 [2.03–7.56] vs. 1.50 [1.50–3.72] pg/ml; *p* = 0.004), although levels of other APPs did not differ between these two subgroups. There were also no significant differences between obese and non-obese subjects concerning other parameters.

Patients with diagnosed metabolic syndrome comprise 27.1% of the study group. Similarly, to obese patients, there were no significant differences concerning the analyzed adipokines and liver function tests in comparison to those without metabolic syndrome. Moreover, comparison between these two subgroups did not demonstrate any differences among APPs (including IL-6). All results are presented in Table 2.

**Table 2:** Comparison of analyzed parameters between patients with and without obesity as well as with and without metabolic syndrome.

Parameters	Non-obese (n = 27)	Obese (n = 32)	*p*	Metabolic syndrome (n = 19)	Without metabolic syndrome (n = 51)	*p*
Chemerin [ng/ml]	256.3 (231.9–287.4)	285.0 (236.1–316.4)	0.16	275.2 (246.7–320.1)	263.7 (234.7–285.9)	0.08
Omentin-1 [ng/ml]	508.5 (334.5–603.1)	449.4 (298.0–678.0)	0.73	441.0 (225.4–600.8)	500.8 (339.6–661.7)	0.67
Vaspin [ng/ml]	0.24 (0.09–0.40)	0.18 (0.12–0.27)	0.30	0.14 (0.07–0.22)	0.17 (0.10–0.30)	0.11
WBC [10^3^/µl]	5.93 (4.68–6.62)	6.24 (5.24–7.50)	0.30	6.16 (5.48–7.43)	5.65 (4.33–6.24)	0.04
HGB [mg/dl]	12.9 (12.4–13.2)	12.8 (11.9–13.9)	0.86	12.9 (12.4–13.0)	12.7 (12.2–13.7)	0.94
PLT [10^3^/µl]	283.0 (205.0–338.0)	253.0 (205.0–335.0)	0.99	314.5 (227.0–403.0)	231.5 (188.0–292.0)	0.003
CRP [mg/l]	5.96 (1.54–7.38)	4.39 (2.98–7.54)	0.90	4.39 (2.13–5.78)	5.88 (1.99–29.8)	0.31
IL-6 [pg/ml]	1.50 (1.50–3.72)	5.32 (2.03–7.56)	0.004	3.42 (1.50–3.98)	2.89 (1.50–7.56)	0.79
Ferritin [µg/l]	175.0 (121.2–258.2)	212.0 (116.0–730.0)	0.11	307.0 (98.2–634.5)	183.5 (123.0–311.0)	0.17
Iron [µmol/l]	20.1 (12.8–23.6)	17.8 (14.3–22.3)	0.52	16.4 (11.3–22.7)	17.4 (11.1–21.7)	0.93
ALT [IU/l]	31.0 (15.0–56.0)	21.0 (17.0–42.0)	0.53	43.0 (26.5–81.0)	32.5 (18.5–52.5)	0.11
AST [IU/l]	22.5 (15.0–45.5)	23.0 (17.5–26.0)	0.94	31.0 (20.2–50.0)	25.0 (17.0–40.2)	0.33
GGT [IU/l]	33.0 (15.5–65.5)	26.0 (18.0–35.0)	0.53	34.0 (18.7–65.0)	32.5 (20.5–63.0)	0.68
ALP [IU/l]	64.0 (50.7–75.7)	57.0 (55.0–76.0)	0.90	61.0 (55.2–79.5)	64.5 (54.0–85.0)	0.65
Bilirubin [µmol/l]	6.09 (3.94–6.92)	6.16 (4.45–7.59)	0.49	5.97 (4.32–7.03)	6.40 (4.70–8.62)	0.21
INR	0.95 (0.93–0.95)	0.95 (0.91–0.98)	0.96	0.97 (0.92–1.04)	0.96 (0.92–1.00)	0.80
Albumin [g/l]	41.0 (37.0–43.0)	40.5 (36.5–43.0)	0.66	40.0 (34.0–42.0)	40.0 (34.7–43.2)	0.44

### Comparison of COVID-19 patients according to infection symptoms: fever, cough, and dyspnea

COVID-19 patients were divided into two subgroups for the presence of fever (body temperature > 38 °C). There was no significant difference in serum chemerin, omentin, or vaspin levels between patients with and without fever. APPs levels did not differ between these two subgroups. There was also no significant difference in respect to liver function tests among patients with and without fever apart from ALP activity which was higher among asymptomatic patients (56.0 [47.0–64.2] vs. 73.5 [57.0–91.0] IU/l; *p* = 0.001). No significant differences were found between patients with and without fever in terms of the other analyzed parameters except for iron concentration, which was higher among patients with body temperature > 38 °C (19.1 [14.3–22.7] vs. 14.3 [8.80–19.7] μmol/l; *p* = 0.04).

A cough was observed in 41 out of 70 patients (59.5%) at the time of hospital admission, while concomitant dyspnea was presented in 20 (28.5%) patients. Patients with a cough had significantly higher body temperature in comparison to the patients without this symptom. There were no significant differences in terms of the adipokines and any of the analyzed laboratory parameters between patients with different temperatures. Surprisingly, COVID-19 patients with intercurrent cough and dyspnea had additionally significantly lower ALT activity as well as significantly lower hemoglobin and fasting glucose levels in comparison to those with an isolated cough. A detailed comparison of analyzed parameters is shown in Table 3.

**Table 3:** Comparison of COVID-19 patients according to infection symptoms: fever, cough, and dyspnea.

Parameters	Cough and dyspnea	Isolated cough	*p*
Chemerin [ng/ml]	246.7 (232.3–279.1)	265.5 (241.8–318.6)	0.09
Omentin-1 [ng/ml]	516.2 (354.6–715.1)	417.8 (264.3–536.3)	0.27
Vaspin [ng/ml]	0.22 (0.07–0.36)	0.15 (0.10–0.26)	0.69
WBC [10^3^/µl]	5.99 (5.11–6.66)	5.93 (4.86–6.97)	1.00
HGB [mg/dl]	13.1 (12.6–13.9)	12.5 (12.0–13.0)	0.03
PLT [10^3^/µl]	279.0 (192.5–330.5)	284.5 (206.5–368.0)	0.67
CRP [mg/l]	5.88 (2.43–11.9)	5.06 (1.86–14.6)	0.88
IL-6 [pg/ml]	3.04 (1.50–11.5)	2.03 (1.50–15.1)	1.00
Ferritin [µg/l]	285.0 (89.3–526.0)	202.0 (141.0–525.0)	0.95
Iron [µmol/l]	15.9 (10.1–21.7)	17.4 (6.77–23.3)	0.57
ALT [IU/l]	25.0 (15.0–37.0)	45.0 (32.5–75.5)	0.003
AST [IU/l]	23.0 (17.2–36.0)	30.0 (20.2–56.2)	0.18
GGT [IU/l]	62.0 (24.0–73.0)	33.5 (18.0–59.0)	0.13
ALP [IU/l]	61.0 (51.5–57.7)	64.0 (54.5–75.5)	0.72
Bilirubin [µmol/l]	6.02 (4.57–7.86)	6.16 (4.70–8.20)	0.98
INR	0.99 (0.95–1.06)	0.93 (0.92–0.95)	0.13
Albumin [g/l]	38.0 (34.0–43.0)	41.0 (37.2–42.0)	0.50

### Comparison of COVID-19 patients with and without gastrointestinal (GI) symptoms

In our study, we differentiated the study group according to the presence of GI symptoms. Inclusion criteria to the group of symptomatic patients were the presence of at least 2 out of 4 symptoms as follows: diarrhea, nausea/vomiting, abdominal pain, dysgeusia. Any of the analyzed adipokines did not differ significantly when compared to COVID-19 patients with and without GI symptoms. However, symptomatic patients had significantly higher iron concentration and lower CRP level in comparison to those without GI problems (22.9 [21.3–23.4] vs. 16.1 [11.7–19.7] μmol/l; *p* < 0.001 and 1.2 [0.77–6.61] vs 5.6 [2.2–21.3] mg/l; *p* = 0.03; respectively). There was no difference in terms of other laboratory parameters between these two subgroups according to GI symptoms.

### Comparison of COVID-19 patients with and without liver injury based on ALT and GGT activities

The patients were also divided into two subgroups based on ALT activity (< 40 and ≥ 40 IU/l). There were no significant differences concerning chemerin, omentin, vaspin levels, and metabolic parameters in groups of patients with different ALT activity. COVID-19 patients with elevated ALT activity presented also a significant increase of other hepatic parameters. No significant elevation of APPs, iron, or any lipid disorders were observed among this subgroup. (Table 4).

**Table 4:** Comparison of COVID-19 patients with different ALT activity.

Parameters	ALT activity < 40 IU/l (n = 36)	ALT activity ≥ 40 IU/l (n = 34)	*p*
Chemerin [ng/ml]	246.7 (232.4–280.9)	275.3 (243.1–315.3)	0.06
Omentin-1 [ng/ml]	503.4 (336.3–669.5)	381.0 (287.6–600.8)	0.24
Vaspin [ng/ml]	0.14 (0.08–0.25)	0.18 (0.14–0.32)	0.20
WBC [10^3^/µl]	5.88 (4.74–6.34)	5.76 (4.40–6.84)	0.89
HGB [mg/dl]	12.8 (12.3–13.8)	12.6 (11.9–13.0)	0.20
PLT [10^3^/µl]	232.0 (189.2–307.7)	260.0 (202.7–342.2)	0.42
CRP [mg/l]	4.79 (1.93–8.18)	3.90 (2.06–25.2)	0.77
IL-6 [pg/ml]	3.35 (1.50–5.87)	1.51 (1.50–7.45)	0.69
Ferritin [µg/l]	176.0 (97.7–322.0)	262.0 (133.2–595.5)	0.12
Iron [µmol/l]	16.5 (11.1–21.7)	16.5 (11.2–22.3)	0.99
AST [IU/l]	18.0 (15.0–23.0)	41.5 (20.0–51.0)	< 0.001
GGT [IU/l]	26.5 (15.0–49.0)	59.0 (32.2–108.2)	0.003
Bilirubin [µmol/l]	5.88 (4.33–6.93)	6.71 (5.02–8.48)	0.03
ALP [IU/l]	56.0 (50.0–69.0)	66.0 (59.5–89.5)	0.002
INR	0.99 (0.92–1.03)	0.95 (0.92–0.97)	0.24
Albumin [g/l]	40.0 (35.0–43.0)	38.5 (34.0–42.0)	0.41

Comparably, no significant difference was observed in patients with elevated GGT activity (≥ 50 IU/l) for adipokines levels. This group of patients presented a statistically significant increase of other hepatic parameters, except for serum bilirubin concentration. Contrarily to the patients with increased ALT, subjects with GGT activity higher than ULN had significantly elevated concentrations of APPs such as CRP or ferritin (Table 5).

**Table 5:** Comparison of COVID-19 patients with and without liver injury based on GGT activity.

Parameters	GGT activity < 50 IU/l	GGT activity ≥ 50 IU/l	*p*
Chemerin [ng/ml]	268.5 (236.8–308.7)	273.3 (237.1–310.9)	1.00
Omentin-1 [ng/ml]	432.4 (312.7–634.1)	521.3 (355.0–680.2)	0.50
Vaspin [ng/ml]	0.15 (0.10–0.25)	0.19 (0.09–0.35)	0.37
WBC [10^3^/µl]	5.98 (5.10–6.61)	4.97 (4.16–6.44)	0.21
HGB [mg/dl]	12.8 (12.3–13.2)	12.7 (11.9–13.5)	0.69
PLT [10^3^/µl]	232.0 (202.2–307.7)	248.0 (199.7–334.2)	0.81
CRP [mg/l]	3.17 (1.75–5.60)	8.07 (3.17–46.8)	0.003
IL-6 [pg/ml]	1.60 (1.50–3.63)	4.79 (1.50–15.1)	0.07
Ferritin [µg/l]	158.0 (98.5–254.5)	351.0 (181.2–697.2)	0.002
Iron [µmol/l]	17.4 (12.0–22.0)	14.3 (8.42–21.4)	0.16
ALT [IU/l]	25.0 (15.2–50.2)	43.0 (33.2–64.5)	0.01
AST [IU/l]	22.0 (15.7–27.7)	37.0 (24.5–49.5)	0.001
Bilirubin [µmol/l]	6.24 (4.33–6.93)	6.13 (4.44–8.34)	0.89
ALP [IU/l]	57.0 (50.7–73.5)	82.0 (64.5–115.2)	< 0.001
INR	0.97 (0.92–0.99)	0.95 (0.92–1.02)	0.72
Albumin [g/l]	40.0 (37.0–44.2)	36.5 (33.0–42.0)	0.01

### Comparison of COVID-19 patients with and without pneumonia

All of the patients at the moment of admission to the hospital were assessed in terms of the presence of clinical or radiological signs of pneumonia. Accordingly, among 23 of 70 patients (32.8%), pulmonary inflammation was diagnosed. When compared COVID-19 patients with and without pneumonia, we did not observe any significant differences in serum chemerin, omentin, or vaspin concentrations. Patients with pneumonia had significantly higher GGT activity (*p* = 0.003), however other liver enzyme activities and bilirubin level remained unchanged. Certainly, markers of inflammation such as CRP, IL-6, or ferritin were significantly elevated among patients with pneumonia. They also presented lower serum total protein and albumin concentrations (Table 6).

**Table 6:** Comparison of analyzed parameters between patients with and without pneumonia.

Parameters	Pneumonia (n = 23)	Without pneumonia (n = 47)	*p*
Chemerin [ng/ml]	260.0 (233.0–281.6)	271.0 (237.9–315.1)	0.24
Omentin-1 [ng/ml]	463.4 (280.2–628.9)	500.8 (355.0–702.3)	0.39
Vaspin [ng/ml]	0.26 (0.10–0.40)	0.15 (0.09–0.24)	0.08
WBC [10^3^/µl]	6.18 (4.76–6.62)	5.70 (4.48–6.36)	0.31
HGB [mg/dl]	12.6 (11.9–13.7)	12.8 (12.3–13.2)	0.66
PLT [10^3^/µl]	301.0 (218.5–405.0)	232.0 (189.7–301.7)	0.02
CRP [mg/l]	6.32 (4.39–40.0)	3.75 (1.77–15.0)	0.04
IL-6 [pg/ml]	5.68 (1.50–17.4)	1.50 (1.50–3.69)	0.006
Ferritin [µg/l]	306.0 (197.0–654.0)	175.0 (91.0–315.0)	0.008
Iron [µmol/l]	17.5 (9.30–22.0)	16.4 (11.7–21.2)	0.79
ALT [IU/l]	31.0 (17.7–45.2)	37.0 (20.7–58.2)	0.33
AST [IU/l]	24.0 (17.5–42.0)	25.5 (18.5–45.5)	0.69
GGT [IU/l]	64.0 (39.0–185.2)	33.0 (20.0–60.0)	0.009
ALP [IU/l]	70.5 (55.0–114.5)	64.0 (54.0–77.0)	0.12
Bilirubin [µmol/l]	6.51 (4.64–8.55)	6.13 (4.45–7.50)	0.51
INR	1.01 (0.95–1.07)	0.95 (0.92–0.99)	0.03
Albumin [g/l]	34.5 (32.0–41.0)	40.0 (37.0–43.7)	0.004

### Comparison of COVID-19 patients requiring and non-requiring Intensive Care Unit (ICU) hospitalization

Among our study group, 15% of patients with diagnosed COVID-19 presented serious clinical condition which required treatment in ICU. No significant differences were found between patients requiring and non-requiring admission to ICU concerning the analyzed adipokines. ICU patients had significantly elevated GGT activity as well as inflammatory markers (WBC count, CRP, IL-6, ferritin) in comparison to the rest of the patients. Patients requiring ICU hospitalization had significantly increased triglycerides, D-dimer, LDH, PLT count, and decreased HDL-cholesterol as well as albumin concentrations. A detailed comparison of analyzed groups was shown in Table 7.

**Table 7:** Comparison of analyzed parameters between patients requiring and non-requiring ICU.

Parameters	ICU (n = 9)	Non-ICU (n = 61)	*p*
Chemerin [ng/ml]	278.1 (233.6–417.7)	271.0 (237.0–309.2)	0.58
Omentin-1 [ng/ml]	593.8 (256.0–652.0)	446.7 (332.7–667.4)	0.78
Vaspin [ng/ml]	0.26 (0.07–0.50)	0.16 (0.10–0.27)	0.61
WBC [10^3^/µl]	8.53 (6.24–10.9)	5.70 (4.42–6.42)	0.003
HGB [mg/dl]	11.3 (10.1–12.6)	12.8 (12.3–13.5)	0.01
PLT [10^3^/µl]	403.0 (273.7–461.2)	232.0 (189.2–308.0)	0.009
CRP [mg/l]	18.2 (5.81–101.0)	4.39 (1.98–11.9)	0.009
IL-6 [pg/ml]	13.5 (6.46–20.9)	1.60 (1.50–5.35)	0.001
Ferritin [µg/l]	765.5 (526.0–1235.0)	208.0 (110.5–381.7)	0.005
Iron [µmol/l]	14.3 (7.55–18.8)	17.4 (11.5–21.8)	0.42
ALT [IU/l]	43.0 (13.2–46.0)	34.0 (20.7–54.2)	0.75
AST [IU/l]	31.0 (19.2–47.2)	25.0 (17.0–43.0)	0.56
GGT [IU/l]	253.0 (103.2–376.5)	33.0 (20.0–62.0)	0.001
ALP [IU/l]	92.0 (58.5–140.2)	64.0 (54.0–80.2)	0.10
Bilirubin [µmol/l]	6.70 (4.89–11.5)	6.14 (4.59–7.77)	0.46
INR	1.03 (0.96–1.08)	0.95 (0.92–1.00)	0.09
Albumin [g/l]	33.0 (27.5–34.7)	40.0 (36.0–43.7)	0.005

### Comparison of COVID-19 patients with different iron and ferritin levels

We also divided patients according to serum iron (≤ 16.8 and > 16.8 μmol/l) and ferritin (≤ 250.0 and > 250.0 µg/l) concentrations. Patients with iron deficiency had statistically significant lower vaspin level (0.13 [0.07–0.22] vs. 0.25 [0.15–0.40] ng/ml; *p* < 0.001). We did not observe any differences regarding chemerin and omentin levels among these patients. The iron deficiency subgroup has also a significantly elevated concentration of APPs (CRP and IL-6), ALP activity as well as total and LDL-cholesterol levels.

Pertaining to patients with elevated and non-elevated ferritin levels, we did not observe differences in any of the analyzed adipokines levels. However, COVID-19 patients with elevated ferritin presented a significant increase of APPs, hepatic parameters (except for ALP activity), and LDH with a contemporaneous decrease of albumin, HDL- and LDL-cholesterol concentrations. The details were described in Table 8.

**Table 8:** Comparison of analyzed parameters between patients with different ferritin as well as iron levels.

Parameters	Ferritin ≤ 250 µg/l (n = 36)	Ferritin > 250 µg/l (n = 28)	*p*	Iron ≤ 16.8 µmol/l (n = 32)	Iron > 16.8 µmol/L (n = 32)	*p*
Chemerin [ng/mL]	255.9 (233.0–417.7)	279.7 (245.5–308.3)	0.25	274.6 (234.5–307.0)	264.9 (236.8–314.9)	0.89
Omentin-1 [ng/mL]	470.9 (298.0–675.9)	463.4 (355.0–603.1)	0.94	455.0 (300.8–671.6)	506.0 (355.0–649.7)	0.90
Vaspin [ng/mL]	0.17 (0.12–0.28)	0.16 (0.09–0.28)	0.64	0.13 (0.07–0.22)	0.25 (0.15–0.40)	< 0.001
WBC [10^3^/µL]	5.70 (4.48–6.68)	5.73 (4.30–6.03)	0.27	5.48 (4.76–6.06)	6.01 (4.30–6.68)	0.62
HGB [mg/dL]	12.7 (12.3–13.4)	12.9 (12.4–13.0)	0.95	12.7 (12.2–13.1)	12.8 (12.4–13.9)	0.31
PLT [10^3^/µL]	253.0 (214.0–323.7)	231.0 (186.2–360.0)	0.43	227.0 (202.2–265.2)	290.0 (203.5–347.7)	0.05
CRP [mg/L]	2.63 (1.35–5.60)	6.04 (3.45–36.0)	0.001	12.6 (4.21–38.7)	2.77 (1.21–5.13)	< 0.001
IL-6 [pg/mL]	1.60 (1.50–3.91)	5.62 (1.50–16.7)	0.01	5.42 (2.62–16.7)	1.50 (1.50–3.60)	< 0.001
Iron [µmol/L]	17.85 (11.9–21.7)	14.3 (6.05–22.5)	0.20	267.0 (111.0–526.0)	175.0 (110.7–258.2)	0.15
ALT [IU/L]	27.0 (16.2–50.0)	44.5 (31.0–66.0)	0.02	37.0 (20.5–56.7)	28.0 (19.2–48.0)	0.44
AST [IU/L]	20.5 (15.5–28.5)	36.0 (25.0–51.0)	< 0.001	25.5 (21.0–41.0)	23.0 (16.2–44.7)	0.24
GGT [IU/L]	26.0 (15.0–47.2)	62.5 (32.0–117.0)	0.001	50.0 (30.5–175.7)	30.0 (18.7–67.2)	0.05
ALP [IU/L]	64.0 (54.7–79.0)	64.0 (55.0–88.0)	0.89	76.0 (56.0–103.2)	61.0 (54.0–72.0)	0.02
Bilirubin [µmol/L]	6.60 (4.48–8.56)	5.99 (4.77–7.21)	0.59	6.00 (4.48–8.97)	6.32 (4.57–7.86)	0.74
INR	0.96 (0.92–0.99)	0.96 (0.92–1.05)	0.46	0.98 (0.91–1.02)	0.95 (0.93–0.97)	0.78
Albumin [g/L]	41.7 (38.5–44.2)	36.0 (32.5–41.0)	0.001	38.0 (33.2–42.7)	41.0 (35.0–44.0)	0.14

### Comparison of COVID-19 patients with different HOMA-IR value

For further analysis patients were divided into two subgroups with HOMA-IR value ≤ 3 and > 3. Analyzing serum concentrations of chemerin, omentin, and vaspin there was no significant difference between COVID-19 patients with various insulin sensitivity (*p* = 0.70, *p* = 0.05, and *p* = 0.52, respectively). COVID-19 patients with HOMA-IR ≤ 3 had significantly lower AST, GGT and ALP activities in comparison to those with HOMA-IR > 3 (22.0 [17.0–26.7] vs. 33.5 [20.5–51.0] IU/l, *p* = 0.02, 27.0 [14.0–35.0] vs. 71.0 [34.7–266.7] IU/l, *p* < 0.001 and 56.0 [52.2–64.2] vs. 67.5 [61.0–91.0] IU/l, *p* = 0.01; respectively). Other parameters associated with liver function tests (ALT, LDH, total bilirubin, INR, albumin) did not differ between these two subgroups. We also observed significantly lower levels of ferritin and IL-6 between COVID-19 patients with various HOMA-IR (167.0 [105.0–526.0] vs. 474.0 [231.2–834.5] µg/l, *p* = 0.04 and 1.50 [1.50–3.26] vs. 5.19 [1.50–10.45] pg/ml, *p* = 0.01; respectively), although levels of other APPs (CRP, PCT) did not differ between these two subgroups. There were also no significant differences between COVID-19 patients with various insulin sensitivity concerning lipid parameters.

Additional comparison of COVID-19 patients with different insulin sensitivity and control group demonstrated that both patients with HOMA-IR ≤ 3 or > 3 had significantly lower chemerin levels in comparison to control group (264.9 [237.2–315.3] vs. 373.0 [363.1–392.3] ng/ml; *p* < 0.001 and 257.8 [234.4–326.9] vs. 373.0 [363.1–392.3] ng/ml; *p* = 0.004, respectively). With respect to omentin significant decrease was observed only comparing HOMA-IR ≤ 3 COVID-19 subgroup with healthy volunteers (399.7 [261.7–566.7] vs. 814.3 [435.3–1148.5] ng/ml; *p* = 0.01), while there was no difference with respect to COVID-19 patients with HOMA-IR > 3 and control group (593.8 [436.7–706.2] vs. 814.3 [435.3–1148.5] ng/ml; *p* = 0.10).

### Results according to lipid disorders

We observed that the vaspin concentration was significantly increased in COVID-19 patients with hypercholesterolemia, increased LDL-cholesterol and hypertriglyceridemia when compared to those with normal lipids levels (0.28 [0.16–0.40] vs. 0.12 [0.08–0.16] ng/ml; *p* < 0.001; 0.28 [0.17–0.49] vs. 0.14 [0.09–0.21] ng/ml; *p* < 0.001; and 0.22 [0.14–0.35] vs. 0.12 [0.07–0.21] ng/ml; *p* < 0.001). Such an association was not found for chemerin and omentin concentrations. Moreover, the group of patients with higher total and LDL-cholesterol levels was characterized by significantly lower CRP and IL-6 serum concentrations as well as significantly elevated PLT count and iron level.

### Correlations between adipokines and basic laboratory parameters

We also analyzed correlations between serum adipokine concentrations and laboratory results as well as clinical parameters. Vaspin serum levels were negatively associated with fasting glucose concentration (r = [− 0.32], *p* = 0.01), whereas positively with body temperature at admission to the hospital (r = 0.34, *p* = 0.006) and LDL-cholesterol level (r = 0.44, *p* < 0.001).

## Discussion

Adipokines, adipose tissue-derived hormones, are presenting a wide range of local, peripheral, as well as central effects. Over the last few years, the vast numbers of studies show a particularly important role of adipokines in the development of various diseases^16,17^. To the best of our knowledge, this is the first study to assess chemerin, omentin, and vaspin levels in COVID-19 patients.

SARS-CoV-2 infection induces defense reaction in the form of the combined immune response of initial cytokine release and activation of antiviral interferon response followed by immune-cell recruitment. In some cases, viral infection can progress to severe disease due to inordinate and dysregulated immune response^18,19^. SARS-CoV-2 induces excessive and prolonged cytokine/chemokine responses in some infected individuals, known as the cytokine storm. The inflammatory cytokine storm is accompanied by immunopathological changes in the lungs, which secondary results in ARDS. As it was mentioned above, overweight and obesity are scientifically proven risk factors of more severe course and in consequence mortality in COVID-19^5–7^. Similarly, patients with T2DM are more prone to develop serious COVID-19 disease and complications such as ARDS and death^8^. This information seems to be crucial for us in the context that the same chronic conditions are directly correlated with fluctuations in analyzed adipokines.

Up to this date, little published research was done analyzing the influence of chemokines or adipokines on the development of SARS-CoV-2 infection. Van der Voort et al.^20^ performed a cross-sectional study measuring serum leptin levels in SARS-CoV-2 virus-infected patients with respiratory failure to investigate if leptin may play a pivotal role in patients with severe SARS-CoV-2 symptoms. SARS-CoV-2 patients admitted to the ICU characterized by hyperleptinemia and implicated a central role of adipose tissue on the pathophysiology of respiratory failure. According to this paper, excessive adipose tissue and leptin production may drive the development of respiratory failure and ARDS in SARS-CoV-2 infected patients.

Our study for the first time showed significantly lower levels of serum chemerin in COVID-19 patients. This fact clearly indicates the crucial role of chemerin in COVID-19 pathogenesis. On the other hand, chemerin serum levels were not associated with the presence of pneumonia, pulmonary or GI symptoms, liver injury, obesity, and metabolic syndrome as well as the severity of infection based on the necessity of admission to ICU. Previous studies presented the pleiotropic role of chemerin in diverse biological processes including immune response regulation and inflammation^21^. It has been proven that increased plasma chemerin is involved in the pathophysiology of various inflammatory diseases^22–27^. Several previous publications also indicated a correlation between circulating chemerin and such markers of inflammation as high-sensitivity C-reactive protein (hs-CRP), IL-6, and tumor necrosis factor α (TNF-α)^28,29^. Moreover, this association appears to be independent of body fat accumulation^30^. This information could indicate the possible role of chemerin in the modulation of the inflammatory process as well as its contribution in inducing extensive inflammatory processes in various inflammatory disorders. It is consistent with our observations since COVID-19 patients with various BMI as well as with or without metabolic syndrome did not present any differences in chemerin concentrations.

What is interesting, chemerin and its role in the physiopathology of viral pneumonia have been already investigated. Bondue et al.^31^ tried to determine the role played by the chemerin/ChemR23 system in the physiopathology of viral pneumonia, using the pneumonia virus of mice (PVM) as a model. According to them, ChemR23^−/−^ mice develop a more severe inflammatory status, higher recruitment of neutrophils and macrophages, higher myeloperoxidase activity, extended macroscopic and microscopic lesions, increased synthesis of pro-inflammatory cytokines (e.g. IL-6) than wild-type mice, resulting in a significant increase in morbidity and mortality rate. In summary, Bondue's study hypothesized that chemerin appears to have anti-inflammatory properties, by acting on ChemR23 expressed by non-leukocytic cells (possibly lung endothelial cells), thereby dampening the inflammatory response promoted by the viral infection.

Since chemerin is perceived as an important factor in the viral inflammatory process some authors indicate the possibility of modulation of this adipokine level in COVID-19 therapy. According to Fioravanti et al.^32^ tocilizumab, an IL-6 receptor antagonist can increase serum levels of adiponectin and reduce circulating leptin, chemerin, plasminogen activator inhibitor-1 (PAI-1), and fibrinogen. It appears that if tocilizumab can reduce circulating chemerin, we can think of this as a mechanism to treat cytokine storms and reduce the risk of thrombosis in patients with COVID-19, although this mechanism certainly needs further investigation to be proved. Our results showed a decrease in chemerin concentration in COVID-19 patients despite the lack of tocilizumab treatment, which indicates its possible anti-inflammatory properties similar to Bondue's study^31^. We also hypothesize that lower chemerin levels could influence disease course and be associated with the necessity of hospitalization due to SARS-CoV2 virus infection, even though we did not observe any differences of these adipokine concentrations between patients with and without pneumonia or hospitalized in ICU. A small group of subjects requiring ICU admission may have interfered with our final results. Furthermore, a decrease in chemerin concentration was not associated with IR indicating that glucose disorders did not influence adipokine level. Equally, chemerin level was independent of liver injury in COVID-19 patients. The above results suggest a direct influence of SARS-CoV2 and the subsequent inflammatory response elicited by the virus on chemerin secretion.

Our study, also for the first time showed significantly lower levels of serum omentin in COVID-19 patients. These findings seem to be consistent with the information presented in the literature, which indicates the anti-inflammatory properties of omentin. The research by Yin et al.^33^ showed a significant decrease of serum omentin level in patients with inflammatory bowel disease (IBD) compared to healthy subjects, with even more evident decrease in those with active disease. According to Rao et al*.,* omentin-1 could potently inhibit TNF-α-induced production of IL-1α, IL-1β, and IL-6, thereby this adipokine is probably able to inhibit the activated macrophages to secrete pro-inflammatory mediators^34^. The anti-inflammatory effects of omentin were also confirmed in chronic hepatitis C patients (CHC)^35^. Another publication also indicates that omentin could reduce the activation of nuclear factor kappa-light-chain-enhancer of activated B cell (NF-kB), and therefore deplete the synthesis of the inflammatory cytokines^36^. The above information implies the possible role of omentin down-regulation in the development of cytokine storm in SARS-CoV2 infection, which are supported by the results of our study, which showed a significant decrease of omentin level among COVID-19 patients. Moreover, this reduction is independent of such factors as metabolic disorders, lipid levels, BMI, respiratory symptoms, or liver injury, implying the direct influence of COVID-19 infection on omentin secretion. A decrease in adipokine concentration was possibly associated with requiring hospitalization. Additional observation of increased omentin concentration among COVID-19 patients with intercurrent IR defined as HOMA-IR > 3 may indicate that its elevation is a compensatory mechanism improving insulin sensitivity.

In the view of the COVID-19 pandemic, the study of Qi and colleagues^37^ investigating the role of omentin in LPS-induced ARDS seems to be intriguing. Compared with the healthy controls, the plasma omentin levels were lower in patients with ARDS. Moreover, the survivors maintained higher concentrations of omentin in comparison to non-survivors. The circulating omentin concentrations negatively correlated with WBCs and PCT levels in patients with ARDS. To assess the effects of increased circulating omentin levels on pulmonary injury response, lung histological examination and ultrastructure pathological examination were performed in mice models treated with an adenoviral vector expressing omentin (Ad-omentin). Ad-omentin protected against LPS-induced ARDS by alleviating the pulmonary inflammatory response and endothelial barrier injury in mice, accompanied by Akt/eNOS pathway activation. According to our study, there was no correlation between omentin and confirmed pneumonia or the necessity of admission to the ICU. Although, as was mentioned earlier a small group of subjects involved in the study may limit data interpretation and needs further investigation to be confirmed.

Another adipokine that was analyzed in our research was vaspin. According to our results, there was no significant difference in vaspin level between COVID-19 patients and controls. Qi and colleagues found vaspin to be protective against LPS-induced ARDS by reversing endothelial cells (ECs) barrier dysfunction via the suppression of inflammation, apoptosis, and ROS production in pulmonary ECs. Moreover, expression levels of the pro-inflammatory cytokines TNF-α and IL-6 were reduced in Ad-vaspin-pretreated mice, whereas expression of the anti-inflammatory cytokine IL-10 was increased^38^. Since vaspin inhibits reactive oxygen species (ROS) and NF-*κ*B signaling pathways, it is believed that vaspin may have a protective role in lung injury, through its anti-inflammatory effect^39^. However, in other publication vaspin plasma concentration was increased in septic patients and correlated with the CRP level^40^. In CHC patients, vaspin was shown to be significantly reduced^41–43^ and positively associated with fibrosis stage. Vaspin was an independent predictor of the severity of liver fibrosis. The further studies are required to assess exact role of vaspin in COVID-19.

Several reports have indicated that more than half of patients with COVID-19 showed varying levels of liver disease^10^. According to our results COVID-19 patients had significantly elevated ALT and GGT activities in comparison to the control group, while there were no significant differences in AST activity or bilirubin level. Moreover, albumin levels were significantly decreased in infected patients. Our observations seem to be consistent with other reports which indicated that abnormal liver function observed in cases of COVID-19, manifesting mainly as isolated elevated serum transaminases and GGT activities^44^. One of the meta-analyses on liver function test (LFT) abnormalities provided an accumulated elevation of AST in 33.3% and ALT in 24.1% of cases^45^. In our study, we have been also investigating the association between LFT abnormalities and the course of infection. Patients with pneumonia had significantly higher GGT activity, however other liver enzymes and bilirubin level remained unchanged. Moreover, COVID-19 patients with intercurrent cough and dyspnea had significantly lower ALT activity compared to patients with isolated cough. Contrarily, Cai and colleagues^46^ as well as Wang and colleagues^47^ presented a significantly higher frequency of cough as COVID-19 initial symptoms among patients with elevated liver enzymes. Surprisingly, the presence of GI symptoms did not influence LFT. It has been suggested that there might be a certain relationship between LFT abnormalities and the severity of COVID-19. In our study ICU patients had significantly elevated GGT and LDH activity. According to Cai et al.^46^ patients with abnormal liver test results, especially in hepatocyte or mixed type, had significantly higher risks of developing severe pneumonia. Several studies performed on Wuhan patients presented that liver injury rates were increased in ICU patients and non-survivors, suggesting that liver injury is most likely to occur in critically ill cases^48–50^. Vespa's study^51^ found ALP activity > 150 IU/l the only predictive factor associated with deterioration.

Taking into consideration the above data it is obvious that LFTs alterations are common in hospitalized patients with COVID-19. The etiology of liver injury is probably multifactorial and associated with drug-induced liver injury and secondary liver injury induced by systemic inflammatory response syndrome or hypoxia. It is still unclear if laboratory LFTs abnormalities have any prognostic value on the COVID-19 course.

Evaluation of LFTs only at admission to the hospital as well as lack of patients with advanced liver disease in the study group are factors that impede comparison of our results with other findings.

Previous studies confirmed that overweight and obesity are one of the most common and prevalent conditions which are correlated with hyperferritinemia^52,53^. On the other hand, it is confirmed that excessive adipose tissue, especially visceral adipose tissue promotes a low-grade inflammatory environment within the body^54^. According to a recent study, ferritin is a marker of inflammation rather than iron status in overweight and obese individuals. Being an acute phase reactant, a high ferritin level secondary to subclinical inflammation in overweight and obese people^55^. Since adipose tissue is undoubtedly a significant endocrine organ we tried to discover if higher plasma ferritin levels correlate with analyzed adipokines concentrations, but this association was not proved.

Since metabolic disorders seem to have colossal impact on different diseases course, including COVID-19, we decided to analyze adipokines levels among patients with varying HOMA-IR values. By that date, only a few studies have been investigating the influence of IR on the course of COVID-19 infection. Most of them emphasized the adverse impact of higher IR on the severity and mortality of COVID-19, suggesting the role of chronic inflammation among these groups of patients^56,57^. Finucane and Davenport^58^ argue that at least in part, a state of IR and elevated insulin levels are driving increased ACE2 expression in lung epithelial cells and, in consequence, aggravating disease severity. On the other hand, COVID-19 can lead to worsening of IR in people with T2DM and T1DM via inducing a pro-inflammatory milieu that can further lead to lowering of insulin sensitivity. Also, SARS-CoV increases serum levels of fetuin-A that has been linked to impaired insulin sensitivity^59^.

Unfortunately, our research has several limitations. First of all, the study group consists of a relatively small number of patients. Secondly, our study did not assess the amount of adipose tissue and mass of muscles that can influence some serum adipokine levels. Furthermore, we included a relatively small number of obese patients. Another serious limitation is the absence of adipokines and other laboratory parameters evaluation during subsequent days of hospitalization, which prevents analyzing adipokine fluctuation with severity of the infection. Subsequent limitation was lack of liver imaging. Also, among our study group there was a disproportion between patient's sexes with dominance of females. Subsequently, the control group had higher median BMI value that COVID-19 patients. Some of these limitations, arise from the fact that our database was created at the very beginning of COVID-19 pandemic. Due to SARS-CoV-2 lock down, that was extremely difficult to recruit and form the control group, which would match ideally the requirements of the study.

## Conclusions

In conclusion, our study revealed, for the first time, serum chemerin and omentin to be significantly decreased in COVID-19 patients compared to healthy controls. Down-regulation of chemerin and omentin levels was independent of obesity, metabolic abnormalities, pulmonary symptoms, and liver function. Since previous publications indicate anti-inflammatory properties of both chemerin and omentin it may suggest that this adipokines deficiency predisposes to a more serious SARS-CoV2 infection requiring hospital admission. The above results indicate SARS-CoV-2 to influence chemerin and omentin levels and thereby up-regulate the development of cytokine storms in SARS-CoV2 infection. On the other hand, there was no relationship between lower adipokines level and frequency of COVID-19 symptoms as well as disease severity based on the necessity of ICU hospitalization. The predictive factors which could predispose to a more severe course of COVID-19, including the presence of pneumonia and ICU hospitalization, were GGT activity, IL-6, and CRP. Pointing to all the results, to determine the exact role of analyzed adipokines and liver injury in SARS-CoV2 infection additional studies are required.

## Methods

### Study population

A total of 70 patients (43 females and 27 males) with a laboratory-confirmed diagnosis of COVID-19 were enrolled. This work was carried out in accordance with the Declaration of Helsinki (2000) of the World Medical Association and was approved by the Ethics Committee of the Jagiellonian University in Cracow (resolution number 1072.6120.157.2020). Subjects provided written informed consent before enrollment to the study. Patients were assessed for eligibility based on a positive reverse-transcriptase–polymerase-chain-reaction (RT-PCR) assay for SARS-CoV-2 from a nasal and/or throat swab. Data on present and past co-morbidities and current medication use were collected. Patients were excluded for the following reasons: hepatitis B virus (HBV) and hepatitis C virus (HCV) infections; human immunodeficiency virus (HIV) co-infection; drug abuse; the presence of neoplastic; thyroid disease; chronic renal failure; mental illnesses; chronic liver disease and cirrhosis based on primary sclerosing cholangitis (PSC), primary biliary cholangitis (PBC), autoimmune hepatitis (AIH) and alcohol cirrhosis (AC). The control group comprised 20 healthy volunteers. The volunteers had no complaints at the time of participation in the study as well as no history of gastrointestinal or chronic liver diseases, smoking and alcohol intake, and systemic diseases. For further analysis, the patients were divided according to their BMI (< 30 and ≥ 30 kg/m^2^) or liver injury based on elevated ALT activity (< 40 and ≥ 40 IU/l) and gamma-glutamyltransferase (GGT) activity (< 50 and ≥ 50 IU/l). Insulin resistance (IR) was calculated according to the homeostasis model assessment for IR (HOMA-IR) by the formula: fasting insulin level (mUI/l) × fasting glucose level (mg/dL)/405. Because HOMA-IR was up-regulated in most of the analyzed patients, for further analysis patients were divided into two subgroups with HOMA-IR value equal to or below 3 and above 3. We also divided patients according to the presence of infection symptoms such as fever, cough, and dyspnea as well as gastrointestinal symptoms (diarrhea, nausea/vomiting, abdominal pain, dysgeusia). Another criterion of the division of the study group was the presence of pneumonia. Assessment of COVID-19 severity was based on the necessity of ICU hospitalization.

### Biochemical and serological assays

Serum samples were obtained from peripheral blood by centrifugation at the moment of hospital admission before any treatment was applied. Chemerin, omentin-1, and vaspin serum concentrations were assessed in duplicate by an immunoenzymatic method with commercially available enzyme immunoassay (EIA) or enzyme-linked immunosorbent assay (ELISA) kits: Human Chemerin ELISA Kit (BioVendor—Laboratorni Medicina a.s., Brno, Czech Republic, with sensitivity 0.1 ng/ml, intra-assay error 6.0% and inter-assay error 7.6%); Omentin-1 ELISA Kit (BioVendor Laboratorni Medicina a.s., Brno, Czech Republic, with sensitivity 0.5 ng/ml, intra-assay error 3.7% and inter-assay error 4.6%. This method included the determination of omentin-1 molecule of full length.); Vaspin ELISA Kit (BioVendor—Laboratorni Medicina a.s., Brno, Czech Republic, with sensitivity 0.01 ng/ml, intra-assay error 7.6% and inter-assay error 7.7%).

The remaining biochemical parameters (such as full blood count, renal function tests, serum ammonia, C reactive protein [CRP]) were measured using routine methods. The upper limit of normal (ULN) of ALT and AST activities was set at 40 IU/l and the ULN gamma-glutamyltransferase (GGT) activity at 50 IU/l.

### Ethics statement

This work was carried out in accordance with the Declaration of Helsinki (2000) of the World Medical Association and was approved by the Ethics Committee of the Jagiellonian University in Cracow (resolution number 1072.6120.157.2020). Subjects provided written informed consent before enrollment to the study.

### Statistical analysis

The data were expressed as median (interquartile range (IQR)). The Shapiro–Wilk test was used to evaluate the distribution. The statistical significance of the difference in studied variables was tested using the Mann–Whitney *U*-test and ANOVA rang Kruskal–Wallis tests for independent groups. Correlations were analyzed with the Spearman rank correlation coefficient. Statistical significance was defined as values of *p* < 0.05. The statistical analysis was performed with STATISTICA 10.0 (StatSoft Polska Sp z o.o., Cracow, Poland).

## Data availability

The data that support the findings of this study are available from the corresponding author, [TR], upon reasonable request.
